# Antibiotic prophylaxis may be still required among transperineal prostate biopsies of diabetics: a cohort study

**DOI:** 10.3389/fmed.2025.1618631

**Published:** 2025-07-04

**Authors:** Feiyue Ma, Yu Zhang

**Affiliations:** Department of Urological Surgery, Xiangshan County First People’s Hospital Medical Health Group, Zhejiang, China

**Keywords:** transperineal prostate biopsy, prostate cancer, urinary tract infections, diabetic patients, antibiotic prophylaxis

## Abstract

**Background:**

Transperineal prostate biopsy (TP-PB) is considered the gold standard for suspected prostate cancer patients. However, the rate of transperineal prostate biopsy-related urinary tract infections (UTIs) has been calculated to be as high as 3%. This study aimed to discuss the incidence of transperineal prostate biopsy -related infections among diabetic patients who underwent antibiotic prophylaxis (AP) or not.

**Methods:**

The monocentric, comparative, observational cohort study was carried out at Xiangshan County First People’s Hospital Medical Health Group, China between January 2021 and January 2023. The study included 246 diabetic men suspected of having prostate cancer who underwent transperineal prostate biopsy. One group was transperineal prostate biopsy with no antibiotic prophylaxis (Group A-no AP, *n* = 120, 48.8%), and the other was given a 3 days of oral antibiotics (Group B-AP, *n* = 126, 51.2%). Data on primary symptoms, urine culture (UC), urinary tract infections incidence, and prostate biopsy -related sequela were gathered 2 weeks following the prostate biopsy.

**Results:**

A total of 246 patients were involved, including 120 in Group A (67.4 ± 7.2 years) and 126 in Group B (68.5 ± 7.0 years) (*p* = 0.215). Prostate-specific antigen (PSA) levels were 16.1 ± 23.8 vs. 15.9 ± 22.3 ng/ml (*p* = 0.942), and the prostate cancer detection rate was 58% vs. 57.5% (*p* = 0.847). The incidence of asymptomatic bacteriuria was significantly higher (8/120, 6.7%) in Group A vs. Group B (1/126, 0.8%) (RR 8.4, 95% CI: 1.1–72.5, *p* < 0.001). Similarly, urinary irritation symptoms occurred in 30/120 (25.0%) vs. 5/126 (4.0%) patients (RR 6.3, 95% CI: 3.0–21.6, *p* < 0.001), fever in 9/120 (7.5%) vs. 1/126 (0.8%) (RR 9.5, 95% CI: 1.3–81.3, *p* = 0.001), and UTIs in 5/120 (4.2%) vs. 1/126 (0.8%) (RR 5.3, 95% CI: 0.63–47.2, *p* = 0.001), respectively. Notably, sepsis was not detected in either group.

**Conclusion:**

Antibiotic prophylaxis could decrease the incidence of transperineal prostate biopsy-related infections among diabetic patients.

## 1 Introduction

Prostate biopsy (PB) is considered the gold standard for diagnosing prostate cancer (PCa), and it is the most frequently conducted procedure in urology departments (1). The conventional approach is often conducted via the transrectal (TR) route. However, TR prostate biopsy (TR-PB) is associated with a relatively high infection rate. Up to 5% of patients who undergo TR-PB require hospitalization due to sepsis (2, 3). Infection has been reported an important cause of death and morbidity among diabetic patients. these patients have a 3- to 4.9-fold risk of kidney infection. Diabetes impairs both innate and adaptive immune system, which impacts the inflammatory response and contribute to increased risk of infections (4, 5). In a prospective randomized trial, Lindert et al. (6) reported a 44% incidence of bacteriuria and a 16% incidence of bacteremia following TR-PB in men with negative preoperative urine cultures.

Transperineal prostate biopsies (TP-PBs) offer comparable cancer detection rates to transrectal biopsies and can be administered under local anesthesia in an outpatient setting (7). More importantly, TP-PB exhibits a lower risk of infection and better sampling advantages than does TR-PB. This approach has gradually gained widespread adoption in clinical practice (7, 8).

Recent investigations into TP-PB, both with and without antibiotic prophylaxis (AP), have reported infection rates that are not significantly different (1, 8). A systematic review and meta-analysis of eight non-randomized studies revealed no impact of AP on infection rates, fever occurrence, sepsis incidence, or readmission rates after TP-PB (9). Despite the relatively low risk of TP-PB-related infection, completely failing to use antibiotics remains challenge for the susceptible population (10, 11). A prophylactic antibiotic therapy was needed before prostate biopsy without making a clear description between the different techniques in the 2021 European Association of Urology (EAU) Guidelines. For the 2024 guidelines on urological infections, AP was recommended for TR-PB. There remains a controversy in both guidelines regarding the necessity of AP for TP-PB (12–14). Moreover, type 2 diabetes is one of the susceptible conditions that leads to a higher risk of infective complications. It is unclear AP is needed among type 2 diabetic patients following TP-PB.

This study aimed to evaluate the incidence of TP-PB-related infections among type 2 diabetic patients who underwent AP.

## 2 Materials and methods

### 2.1 Study design

This was a single-center, comparative, observational cohort study carried out between January 2021 and January 2023 was conducted at Xiangshan County.

First People’s Hospital Medical Health Group, China (Registration number 2500095587). We collected 246 patients diagnosed with type 2 diabetes with a clinical suspicion of PCa and prepared them for TP-PB at Xiangshan County First People’s Hospital medical health group. The diagnosis of type 2 diabetes relies on the 1990 WHO criteria. Patients with plasma HbA1c levels (6.5%–12%) were included (15). All consecutive adult diabetic patients with TP-PB were prospectively included and provided informed consent. The included patients received the TP-PB for the first time and only once. Patients with a history of recurrent UTIs or recorded UTIs were excluded. Patients with AP were compared with those without AP to analyze TP-PB-related infections. Given the absence of specific guidelines for AP in diabetic patients undergoing TP-PB, allocation of prophylaxis was determined through subjective decision-making of urologist and/or patients’ requests. The AP scheme followed the European Association of Urologists (EAU) guidelines, and cefixime (400 mg once per day for 3 days) was used starting 24 h before TP-PB (16). This study was approved by the Ethics Committee of Xiangshan County First People’s Hospital Medical Health Group.

Before biopsy, all patients underwent urine culture, with follow-up culture performed 14 days after TP-PB. Three weeks after TP-PB, patients were assessed in the outpatient clinic to evaluate TP-PB-related complications. These parameters included gross hematuria, urinary retention, urethrorrhagia, hematospermia, pre- and postoperative total leukocyte counts, postoperative fever (defined as a temperature exceeding 38°C), postoperative urinary tract infection (significantly elevated white blood cell counts in urine analysis, > 5 per high-power field, possibly accompanied by symptoms such as painful micturition bladder, suprapubic, or renal pain, urinary frequency, urgency, dysuria, cloudy and foul-smelling urine, and fever), and sepsis (characterized by systemic inflammatory response syndrome and organ dysfunction).

### 2.2 Biopsy procedure

All TP-PB procedures were performed by experienced urologists in an outpatient setting. The patients received an enema and fasted before the TP-PB. The dorsal lithotomy position with gynecological heel stirrups was applied throughout the procedure. Local anesthesia (lidocaine hydrochloride 1% 10 ml) was administered in the ventral prostatic apical region after perineal and perianal skin disinfection (10% povidone-iodine solution). TP-PB was conducted with a color ultrasound diagnostic system (Philips EPIQ5) combined with a disposable automatic biopsy needle (18G*20 cm, Kanaiwei Medical Technology, Zhejiang, China). The needle was inserted via a single hole in the middle of the perineum, 1.5 cm from the anus. The number of cores depended on the prostate volume, MRI-based fusion biopsy, and saturation biopsy.

### 2.3 Statistics

All the statistical analyses were performed via R software (version 4.1.0). We utilized a conservative estimate of 5% infection rate in the non-prophylaxis group and 1% in the prophylaxis group and the sample size was calculated out for 120 patients per group provided 80% power to detect a difference in infection rates, with a two-sided α of 0.05. Continuous variables are expressed as the mean ± standard deviation (SD). Categorical variables are presented as numbers and percentages. The normality of continuous variables was assessed via the Shapiro–Wilk test. Baseline characteristics were compared between groups via Student’s *t*-test for normally distributed continuous variables, the Mann–Whitney U test for non-normally distributed continuous variables, and the chi–square test or Fisher’s exact test for categorical variables.

For the primary outcome analysis, infection-related outcomes (urinary irritation symptoms, fever, sepsis, and UTIs) were compared via the chi-square test for frequencies > 5 and Fisher’s exact test for frequencies ≤ 5. Risk ratios (RRs) with 95% confidence intervals (CIs) were calculated for categorical outcomes. For the secondary outcome analysis, WBC counts were compared via Student’s *t*-test after confirming a normal distribution. Multiple logistic regression was performed to adjust for potential confounding factors: age, BMI, duration of diabetes, and HbA1c levels. Adjusted odds ratios (ORs) with 95% CIs were calculated.

This statistical methodology follows the CONSORT guidelines for reporting randomized clinical trials and provides a comprehensive approach to analyzing the effectiveness of antibiotic prophylaxis in transperineal prostate biopsy among diabetic patients. The methods were chosen to ensure robust analysis while accounting for potential confounders and maintaining statistical validity.

## 3 Results

A total of 246 consecutive patients were analyzed. A total of 120 patients received TP-PB without AP, and 126 patients were administered AP before the procedure. The baseline data of the enrolled patients are presented in Table 1. In both cohorts, there were no statistically significant differences in terms of age, body weight, body mass index (BMI), systolic pressure, diastolic pressure, glycated hemoglobin a1c (HbA1c), low-density lipoprotein (LDL), estimated glomerular filtration rate (eGFR), prostate-specific antigen (PSA), prostate volume, biopsy cores, or duration of diabetes *(p* > 0.05, *t*-test). Additionally, white blood cell (WBC) counts before TP-PB were within the normal range in the two cohorts, with no statistically significant differences (*p* > 0.05, *t*-test).

**TABLE 1:** Baseline data of the enrolled patients.

	Cohort A-no AP (*n* = 120)	Cohort B-with AP (i = 126)	*P*-value
Age (years)	67.4 ± 7.2	68.5 ± 7.0	0.215
Body weight (kg)	70.3 ± 7.4	68.0 ± 8.0	0.187
BMI (kg/m^2^)	26.6 ± 4.4	27.0 ± 2.4	0.342
Systolic pressure (mmHg)	134.35 ± 20.14	136.27 ± 18.85	0.425
Diastolic pressure (mmHg)	74.34 ± 14.21	74.48 ± 15.13	0.938
HbA1c concentration (%)	7.9 ± 0.9	8.1 ± 1.2	0.124
LDL (mmlo/L)	3.76 ± 0.63	3.78 ± 0.74	0.815
eGFR (mL/min)	90.6 ± 16.1	90.4 ± 17.6	0.924
PSA (ng/ml)	16.1 ± 23.8	15.9 ± 22.3	0.942
Prostate volume (ng/ml)	52.5 ± 10.6	51.9 ± 8.9	0.632
Biopsy cores (i)	14.5 ± 1.8	14.7 ± 2.3	0.437
Duration of diabetes (years)	8.8 ± 2.4	8.7 ± 2.6	0.756
Pre-WBC (10∧9/L)	7.11 ± 1.82	7.09 ± 1.81	0.932

BMI, body mass index; LDL, low density lipoprotein; eGFR, estimated glomerular filtration rate; PSA, prostate-specific antigen; WBC, white blood cell.

Table 2 shows the non-infectious indicators of the two groups. The only significantly different domain was asymptomatic bacteriuria (Figure 1a, 8 in cohort A vs. 1 in cohort B, *p* < 0.05, 95%CI: 1.1–72.5, chi-square test), whereas other domains, including the prostate cancer detection rate (*p* > 0.05, chi-square test), postoperative hematuria (*p* > 0.05, chi-square test), and urinary retention (*p* > 0.05, Fisher’s exact test), were not significantly different.

**TABLE 2:** Reported non-infectious indicators of the two groups.

	Cohort A-no AP (*n* = 120)	Cohort B-with AP (*n* = 126)	*P*-value
Prostate cancer detection rate	70 (58.3)	72 (57.1)	0.847
Asymptomatic bacteriuria (*n*, %)	8 (6.7)	1 (0.8)	< 0.001
Postoperative hematuria (*n*, %)	20 (16.7)	18 (14.3)	0.598
Urinary retention (*n*, %)	2 (1.7)	1 (0.8)	0.614

**FIGURE 1:** Statistical analysis of the clinical outcomes of theand two groups. **(a)** Asymptomatic bacteriuria. **(b)** Urinary irritation symptoms. **(c)** Fever and urinary tract infections (UTIs) incidence. **(d)** White blood cell (WBC) levels.

Table 3 summarizes the TP-PB-related infectious indicators. The incidence of lower urinary tract symptoms (Figure 1b, *p* < 0.05, 95% CI: 3.0–21.6, chi-square test), fever (Figure 1c, *p* < 0.05, 95% CI: 1.3–81.3, chi-square test), and UTIs (Figure 1c, *p* < 0.05, 95% CI: 0.63–47.2, chi-square test) in Cohort A was greater than that in Cohort B. We have analyzed the microbiological profiles of patients who developed UTI. Among the 6 confirmed UTI cases (5 in Group A, 1 in Group B), urine cultures yielded: *Escherichia coli* in four patients (66.7%), *Klebsiella pneumoniae* in one patient (16.7%), and *Enterococcus faecalis* in one patient (16.7%). All *E. coli* isolates demonstrated susceptibility to cefixime (MIC ≤ 1 μg/mL), while the *K. pneumoniae* isolate showed intermediate susceptibility. Compared with that in Cohort B, the WBC count was significantly greater in Cohort A after TP-PB (Figure 1d, *p* < 0.05, Student’s *t*-test). Notably, sepsis was not detected in either group.

**TABLE 3:** Summary of the transperineal prostate biopsy (TP-PB)-related infectious indicators.

	Cohort A-no AP (*n* = 120)	Cohort B-with AP (*n* = 126)	*P*-value
Urinary irritation symptoms (*n*, %)	30 (25.0)	5 (4.0)	< 0.001
WBC (10∧9/L)	11.46 ± 2.59	8.57 ± 2.56	< 0.001
Fever (*n*, %)	9 (7.5)	1 (0.8)	0.001
UTIs (*n*, %)	5 (4.2)	1 (0.8)	0.001
Sepsis (*n*, %)	0	0	–

WBC, white blood cell; UTIs, urinary tract irritation symptoms and pyuria accompanying positive urine culture.

## 4 Discussion

According to the 2024 Guidelines of the EAU, TP-PB has a lower risk of infectious complications than does TR-PB, and it is strongly recommended for high-risk patients (17). A shift to TP-PB for obtaining pathology specimens suspicious of CaP has taken place. Several studies have reported that TP-PB rarely causes sepsis without AP (18, 19). In one retrospective single-center cohort study, Sigle et al. (20) reported that TP-PB without AP is a safe procedure and results in fewer TP-PB-related infections, such as fever and sepsis. While TP-PB may curtail infection, it still induces infection ranging from approximately 0.10%–3% (10). One study reported that several factors, including diabetes, bacterial prostatitis, history of urinary retention, history of urinary infection, and number of cores, are associated with TP-PB-related infectious complications. The study revealed that diabetes was independent risk factor of TP-PB-related infectious complication. There was no exact reason for diabetes increasing the risk of the infectious complications (10, 11). In this study, we evaluated the effect of AP on diabetic patients with TP-PB.

In our study, there were eight cases of asymptomatic bacteriuria (6.7%), 30 cases of urinary irritation symptoms (25%), nine cases of fever (7.5%), and five cases of UTIs (4.2%) in the group without AP. None of the patients in either cohort developed sepsis. Compared with Cohort B, candidates without AP had a greater WBC count and were more likely to develop TP-PB-related infectious complications. This finding is inconsistent with recent findings (1, 2, 9).

A retrospective study carried out on 326 consecutive patients demonstrated that the routine use of antibiotics with TP-PB does not affect morbidity rates. However, the study did not perform subgroup analysis. Patient demographics were based on ethnicity, not basic medical history (1).

Pirola et al. (2) reported that the incidence of UTIs and bacteriuria in TP-PB is not correlated with AP. He suggested that AP is not needed in TP-PB patients. Notably, few diabetic patients were included in this study, and the outcome could not be used to determine the effect of AP on the TP-PB among diabetic patients (2).

The results from a systematic review also confirmed that fever, infection rate, readmission rate, and sepsis after TP-PB were not significantly different between the AP group and the non-AP group (9, 21). However, this meta-analysis neither performed heterogeneity analysis nor selected a specific population for analysis.

One randomized controlled trial demonstrated that patients who underwent TP-PB with no antibiotic use were non-inferior to those who received AP (3). The RCT and prior studies have suggested a low incidence of TP-PB-related infections, regardless of the use of APs (3, 5, 22). However, these studies were underpowered and had limitations for the populations (3, 5, 22).

The novelty of this study lies in the special population of diabetic patients. Owing to its susceptibility to infection, AP is vital for diabetic patients undergoing TP-PB. However, there are several limitations to this study. First, the two cohorts were only from a single center, and the number of patients was small. Moreover, we did not collect data on the medication history of diabetes and did not determine the correlation between diabetes and TP-PB-related infections. Finally, we excluded other high-risk factors and reduced the complexity of the data, so we are uncertain about the role of AP in TP-PB-related infection under complex conditions.

## 5 Conclusion

Thus, diabetic patients receiving TP-PB may need AP. It could decrease the incidence of TP-PB-related complications, such as asymptomatic bacteriuria, urinary irritation symptoms, fever, and UTIs. AP could still be needed in TP-PB candidates with a high risk of infections in the future.

## Data Availability

The raw data supporting the conclusions of this article will be made available by the authors, without undue reservation.
